The article "Strychnos pseudoquina modulates the morphological reorganization of the scar tissue of second intention cutaneous wounds in rats" was retracted in 2025. Reasons: duplicated images; overlap with earlier publications; original data or images not available; concerns about the images.

# *Strychnos pseudoquina* modulates the morphological reorganization of the scar tissue of second intention cutaneous wounds in rats

**DOI:** 10.1371/journal.pone.0195786

**Published:** 2018-04-12

**Authors:** Mariáurea Matias Sarandy, Lyvia Lopes Miranda, Luciana Schulthais Altoé, Rômulo Dias Novaes, Virgínia Vinha Zanuncio, João Paulo Viana Leite, Reggiani Vilela Gonçalves

**Affiliations:** 1 Department Animal Biology, Universidade Federal de Viçosa, Viçosa, Minas Gerais, Brazil; 2 Institute of Biomedical Sciences, Department General Biology, Universidade Federal de Viçosa, Viçosa, Minas Gerais, Brazil; 3 Department of Structural Biology, Universidade Federal de Alfenas, Alfenas, Minas Gerais, Brazil; 4 Department of Medicine and Nursing, Universidade Federal de Viçosa, Viçosa, Minas Gerais, Brazil; 5 Department of Agricultural Biochemistry, Universidade Federal de Viçosa, Viçosa, Minas Gerais, Brazil; Ohio State University, UNITED STATES

## Abstract

Natural substances are used in folk medicines to treat injuries. *Strychnos pseudoquina* has scarring, antipyretic, and antimalarial actions. The present study aimed to analyze the effect of *S*. *pseudoquina* on cutaneous wound healing in rats. The *S*. *pseudoquina* extract was submitted to phytochemical prospection. The levels of flavonoids and total phenolic compounds in the extract were 50.7 mg/g and 2.59 mg/g, respectively. Thirty Wistar rats were individualized in cages with food and water *ad libitum* (registration no. 730/2014). After anesthesia, three circular wounds (12mm diameter) were made in the animals, which were randomly separated into five treatments: Sal, saline; VO, ointment vehicles (lanolin and Vaseline); SS, positive control (silver sulfadiazine 1%); LE 5, freeze-dried extract 5%; and LE 10, lyophilized extract 10%. The animals were treated with the ointment daily for 21 days. Every seven days, the area and the rate of wound contraction were evaluated. Tissue samples were removed for histopathological analysis of the number of mast cells, elastic and collagen fibers, and biochemical analyses, quantification of malondialdehyde (MDA), carbonylated proteins (PCN), superoxide dismutase (SOD), catalase (CAT), transforming growth factor β (TGF-β), Interleukin 10 (IL-10) and tumor necrosis factor (TNF). The number of mast cells, collagen and elastic fibers in the rat wounds were higher in the treatments with the plant. The extract also stimulated the activity of antioxidant enzymes, particularly SOD, presenting high levels, and maintained low levels of PCN. The TGF-β and IL-10 concentration was higher in the LE5 and LE10 treatment of the extract than in the Sal, OV and SS treatments on day 7. The ointment based on *S*. *pseudoquina* closed the wound faster and accelerated wound healing in animals.

The article "Strychnos pseudoquina modulates the morphological reorganization of the scar tissue of second intention cutaneous wounds in rats" was retracted in 2025. Reasons: duplicated images; overlap with earlier publications; original data or images not available; concerns about the images.

## Introduction

Wounds with proximal cut edges, common in surgical procedures, are termed first intention [1]. Secondary-intention wounds present tissue loss and a slower healing process due to the need for new tissue growth [2]. Lack of healing leads to suffering for the patients and a negative impact on the physical, social, emotional development, and economic aspects of their lives. Failures or delays in the healing process may be related to patient characteristics, such as age and medical condition [3]. Malnutrition, diabetes mellitus, immunodeficiency and venous stasis may delay the healing process [4,5].

Cytokines and cells can heal cutaneous wounds faster [6,7]. This process includes the inflammatory, proliferative and tissue maturation or remodelling phases [8,9]. However, changes in any of these phases may lead the cutaneous lesion to become chronic [10,11].

Phagocytes, recruited to the lesion site, perform a respiratory explosion, releasing free radicals and reactive oxygen species (ROS), as defense against pathogens during the skin repair process, especially in the inflammatory phase [12]. The continuous production of ROS causes oxidative stress, which leads to degenerative changes and increases tissue damage, thus forming a fragile and scarcely resistant scar [13]. Detoxification of cells by the activation of antioxidant defense systems, especially superoxide dismutase (SOD) and catalase (CAT) enzymes, guarantees a harmonious process of tissue repair [14,15].

Cells recruited in the inflammatory phase release cytokines and growth factors that mediate cell migration and differentiation in the proliferative phase of cutaneous repair [16]. The efficient and infection-free scarring process depends on factors, such as tumor necrosis factors alpha (TNF-α), platelet-derived growth factor (PDGF), fibroblast growth factor (bFGF), transforming growth factor β (TGF-β) and epithelial growth factor (EGF) [17].

Weak and brittle type III collagen is replaced by strong, tensile-resistant type I collagen in the last stage of the healing process, when fibroblasts, which synthesize the matrix components, predominate and the number of blood vessels decreases [18,19]. Modulating agents stimulate the healing process of cutaneous wounds [7,20,21]. Plants stand out in folk medicine [22,23], including *Strychnos pseudoquina* St. Hil. (Loganiaceae), native to the Brazilian *cerrado*. Stem bark is the most commonly used part of this plant [24–26]. Barks and leaves are also used as antipyretics, antimalarials and in the treatment of disorders of the gastrointestinal system [27–29]. Extracts from *S*. *pseudoquina* have protected the gastric mucosa of mice against lesions caused by Anti-inflammatory drugs and acidic ethanol solutions, reducing pre-established lesions and increasing the cellular and vascular proliferation of the injured region [30].

The article "Strychnos pseudoquina modulates the morphological reorganization of the scar tissue of second intention cutaneous wounds in rats" was retracted in 2025. Reasons: duplicated images; overlap with earlier publications; original data or images not available; concerns about the images.

This study aimed to analyze the morphological reorganization and oxidative status in the healing process of secondary intention cutaneous wounds in rats treated with *S*. *pseudoquina* ointment.

## Materials and methods

### Plant material collection

Samples from *S*. *pseudoquina* were collected in the city of Rio Verde, Goiás, Brazil, dried in an oven at 40 degrees Celsius and sprayed with knife mills. Exsicates of *S*. *pseudoquina* were deposited in EPAMIG-BH herbarium (PAMG number 57079). These samples were dehydrated, pulverized with ethyl alcohol (95%), which was used as the extracting solvent, and subjected to a percolation extraction process. The extract from *S*. *pseudoquina*, after exhaustive extraction, was concentrated in a rotary evaporator for the removal of the solvent and lyophilized so as to obtain the dried extract [31]. The phytochemical components of the extract were analyzed by chromatography on plates covered with silica gel GF 254 (Merck, Darmstadt, Germany) with different mobile phases and detection reagents [32].

### Preparation of the formulation and standard used

The *S*. *pseudoquina* lyophilized extract was mixed in a ceramic mortar and pestle and emulsified in lanolin at concentrations of 5% and 10% (v / v) for the preparation of the ointment. Silver sulfadiazine cream (1%) from Rexin Pharmaceuticals Pvt Ltd. was used as the standard drug (positive control).

### Animals

Thirty healthy male Wistar rats (*Rattus norvegicus*) with five weeks of life (198.25 ± 26.11g), fed on a standard commercial diet, were obtained from the Central Biotério of the Universidade Federal de Viçosa and separated in cages, cleaned daily and kept under environmental conditions (Temperature: 22 ± 2°C, humidity: 60 to 70%, and light / dark cycle: 12/12 h). The procedures were approved by the animal use ethics committee—UFV (registration no. 730/2014).

### Realization of surgical wounds

The rats were anesthetized by intraperitoneal injection of ketamine (60 mg/kg body weight) and xylazine (10 mg/kg body weight). For analgesia and to avoid the suffering of the animals was applied by intraperitoneal route Pentobarbital (30mg / kg of animal weight). After anesthesia, three circular 12 mm diameter wounds were made in the dorso-lateral region of each rat by secondary intention, with surgical excision of the skin and subcutaneous cellular tissue using a metallic puncture. The area of the wounds was marked with violet crystal and measured with an analog caliper (Mitutoyo Sul Americana Ltda^®^, São Paulo, Brazil). The animals' skin was removed until the dorsal muscular fascia was exposed to control the depth of the surgical incision [33].

The article "Strychnos pseudoquina modulates the morphological reorganization of the scar tissue of second intention cutaneous wounds in rats" was retracted in 2025. Reasons: duplicated images; overlap with earlier publications; original data or images not available; concerns about the images.

Tissue samples were obtained from different wounds at 7, 14 and 21 days for histological, biochemical and cytokine expression analysis. A tissue sample was removed on the first day of the experiment (F0) and stored for analysis of the uninjured tissue. A sample of the first (F1), second (F2) and third (F3) wounds of each animal was removed on the seventh, 14^th^ and 21^st^ days, respectively.

### Area and rate of wound contraction

The area and rate of contraction of the third wound were evaluated every 7 days using images scanned with 320×240 pixels (24 bits/pixel) obtained by digital camera (W320 Sony, Tokyo, Japan). The wound area was calculated by computerized planimetry using Image-Pro Plus 4.5 (Media Cybernetcs, Silver Spring, USA). The wound contraction index (WCI) was calculated by the ratio: initial wound area (Ao)—area on a given day (AI) / initial wound area (Ao) × 100 [34].

### Experimental design

The animals were randomly separated into five treatments (n = 06/treatment): wounds treated with saline solution at 0.9% (Sal-control); Control wounds treated with 0.6g silver sulfadiazine (1%) (SS); Wounds treated with 0.6g of lanolin cream (OV-ointment vehicle); Wounds treated with *S*. *pseudoquina* extract at 5% concentration (LE 5); Wounds treated with *S*. *pseudoquina* extract at 10% concentration (LE 10). The wounds were cleaned daily with 0.9% saline solution prior to treatment for 21 days. Then, the animals were euthanized by cervical dislocation.

### Histological analysis

The samples collected from the wounds, with tissue from the center of the lesion and part of the tissue adjacent to the edges of the lesions, were fixed in 10% formaldehyde solution buffered in 0.1 M sodium phosphate (pH 7.2), dehydrated in ethyl alcohol, Diaphanized in xylol and immersed in paraffin. Histological sections (4μm thick) were obtained on Leica Multicut® 2045 rotary microtome (Reichert-Jung Products, Germany). These sections were mounted on a histological slide and stained with Hematoxylin and Eosin for the analysis of fibroblasts and blood vessels [35], stained with Sirius Red for the analysis of collagen fibers [36], using toluidine blue for evidence of mast cells and resorcin fuchsin to mark elastic fibers [37]. One in ten cuts was used to avoid repeated analysis of tissue constituents. The slides were visualized and captured in a BX-60® light microscope (Olympus, São Paulo, Brazil) coupled to a QColor-3® digital camera (Olympus, São Paulo, Brazil). Four slides, containing six histological sections, were made per wound and stained. Fifteen images were obtained by random cutting, with resolution of 2048 X 1536 pixels and 20x magnification. Fibroblasts, blood vessels, elastic and collagen fibers and mast cells were counted in scanned images with a grid of 216 intersections associated with the Image Pro-plus 4.5 (Media Cybernetcs®, Silver Spring, USA), a software system for image analysis.

The article "Strychnos pseudoquina modulates the morphological reorganization of the scar tissue of second intention cutaneous wounds in rats" was retracted in 2025. Reasons: duplicated images; overlap with earlier publications; original data or images not available; concerns about the images.

### Biochemical analysis

Tissue samples removed from each wound were immediately frozen in liquid nitrogen (-196°C) and stored in a freezer at -80°C. Extracts from these samples were homogenized in phosphate buffer and centrifuged at -5°C. Peroxidation markers were analyzed on the supernatant. The malondialdehyde (MDA), [38] carbonylated proteins (PCN) [39] levels and the antioxidant enzyme activities were analyzed. Catalase (CAT) [40] was measured by the hydrogen peroxide (H_2_O_2_) and superoxide dismutase (SOD) decomposition rate, following the Siddiqui et al. [41] protocol. Biochemical data was normalized according to the total protein levels in the supernatant [42].

### Analysis of cytokine expression

Scar tissue samples, collected on days seven and 14, were frozen at -80°C, homogenized in PBS 7.4 buffer containing 0.05% Tween and centrifuged at 3500g, for 30 minutes. The TGF-β, IL-10 and TNF levels in the supernatant were analyzed with the use of immunoassay kits, by the ELISA method (Boster Biological Technology Ltd., China), following the manufacturer's recommendations. High affinity polystyrene plates (Corning, New York, USA) were coated with 100 mL/well of monoclonal antibodies, specific to the component to be assayed (capture antibody), diluted in carbonate-bicarbonate buffer 0.1 M (pH 9.6) for 12 hours, at 4°C. Thereafter, these plates were blocked with PBS solution supplemented with 10% inactivated fetal bovine serum (Sigma) for one hour at room temperature. Recombinant compounds (standard curve) and samples of plasma or homogenized scar tissue were added in duplicate to the wells of the plates [31], which were incubated at room temperature for two hours and washed five times with PBS-Tween. Biotin-conjugated (detection antibody) secondary antibodies specific to each component of interest, and associated with avidin-peroxidase were added to the concentrations recommended by the manufacturar. The reaction was developed with tetramethylbenzidine (TMB) and blocked after 20 minutes with 2M sulfuric acid. The reading was performed on a microplate reader (Power Wave X-Bio Tek Instruments, Inc.).

### Statistical analysis

The data was represented by central tendency measures, mean and standard deviation (SD). The data distribution was verified by the D'Agostino-Pearson test and Kruskal-Wallis variables for multiple comparisons. The statistical significance was p <0.05. The data was analyzed with the aid of the GraphPad Prism 5.0® (GraphPad Software Inc., San Diego, Calif., USA) software system.

The article "Strychnos pseudoquina modulates the morphological reorganization of the scar tissue of second intention cutaneous wounds in rats" was retracted in 2025. Reasons: duplicated images; overlap with earlier publications; original data or images not available; concerns about the images.

## Results

### Phytochemical analysis

The Phytochemical prospection of *S*. *pseudoquina* extract indicated the presence of flavonoids and alkaloid phenolics. The rates of flavonoids and total phenolic compounds in the extract were 50.7 mg / g and 2.59 mg/g, respectively.

### Wound area and wound contraction index

The wound area was smaller on days 7, 14 and 21, with 5 and 10% *S*. *pseudoquina*, compared to Sal, OV and SS. The wound contraction rate was higher with 5 and 10% *S*. *pseudoquina* extract, on day seven (Table 1).

**Table 1:** Area (mm^2^) and rate of wound contraction (RWC) (%) in animals treated with *Strychnos pseudoquina* extract at different concentrations.

		Sal	OV	SS	LE (5%)	LE (10%)
Day 0	Area	120.1±10,6	123.5±9.6	125.3±9.5	120±10.1	123.5±10.5
	RWC	0.0±0.0	0.0±0.0	0.0±0.0	0.0±0.0	0.0±0.0
Day 7	Area	112.4±9.9	113.1±9.9	110.6±8.1	90.5±10.3*	70.5±10.7*
	RWC	21.7±7.4	29.5±8.6	27.7±10.0	52.4±8.7*	58.5±9.6*
Day 14	Area	80.0±11.3	65.2±12.9	54.1±10.4	15.9±8.8*	16.8±8.1*
	RWC	64.7±9.3	78.3±7.9	67.9±9.1	79.1±7.5	79.9±5.5
Day 21	Area	5.4±1.4	3.2±1.1	4.43±1.6	0.8±0.07*	0.2±0.05*
	RWC	94.3±5.3	94.0±5.3	94.9±2.6	98.0±1.2	96.7±2.4

Tissue fragments were collected every seven days for 21 days of treatment. Sal: saline 0.9%; OV: ointment vehicle; SS: silver sulfadiazine (1%), LE 5: *S*. *pseudoquina* extract (5%); LE 10: *S*. *pseudoquina* extract (10%). The treatments were applied directly to the wounds for 21 days. F0 = intact tissue; F1, F2, F3 = cicatricial tissue after seven, 14 and 21 days, respectively. * Statistical difference vs. Sal, OV and SS.

### Histopathological results

The number of mast cells was higher in wounds treated with *S*. *pseudoquina* extract at 5 and 10% on days 7 and 21 when compared to the other groups. On day 14, *S*. *pseudoquina* 10% was higher than all the other groups, but LE 5% was only higher than the control groups (Fig 1A). These results can be observed in the photomicrographs 1B and 1C.

**Fig 1:** A- Ratio of mast cells in scar tissue from rats treated with *Strychnos pseudoquina* extract. F0: untreated normal tissue, F1: treated tissue after seven days, F2: treated tissue, after 14 days, F3: tissue treated after 21 days. Sal: saline solution, OV: vehicle, SS: silver sulfadiazine, LE 5: *S*.*pseudoquina* 5%; LE 10: *S*. *pseudoquina* 10%. Data represented as mean ± SD. *^†^ p <0.05, statistical difference between treatments: * vs. Sal and OV, *† vs. Sal, OV and SS (Kruskal-Wallis test). B, C- Photomicrographs of mast cells in the scar tissue treated with *S*. *pseudoquina*, 200X and 400X magnification, Bar = 20μm and 10 μm, respectively.

The article "Strychnos pseudoquina modulates the morphological reorganization of the scar tissue of second intention cutaneous wounds in rats" was retracted in 2025. Reasons: duplicated images; overlap with earlier publications; original data or images not available; concerns about the images.

The ratio of type I collagen fibers was higher with 5 and 10% *S*. *pseudoquina* extract throughout the experimental period. However, on day 14, SS was also higher than the control groups (Figs 2A and 3). On day 7, the ratio of type III collagen was higher in treatments SS, LE5 and LE10 than in controls; and, on day 14, it was higher with *S*. *pseudoquina* extract than with other treatments (Figs 2B and 3). The number of elastic fibers on days 14 and 21 increased in treatments with *S*. *pseudoquina*, at 5 and 10% (Fig 2C). Fig 3 shows collagen deposition throughout the experiment. On day 0, there is a large number of collagen type I fibers (Yellow-Red), since they demonstrate the amount of normal tissue found. On days 7 and 14, there is a reduced number of type I collagen and an increased amount of collagen type III (green), since it represents the granulation tissue. On day 21, it was observed increased type I collagen, mainly in the groups treated with the extract.

**Fig 2:** **Proportion of collagen fibers of type I (A) and III (B) and elastic (C) types in scar tissue of rats treated with *Strychnos pseudoquina* extract**. F0: untreated normal tissue, F1: treated tissue after seven days, F2: treated tissue, after 14 days, F3: treated tissue after 21 days. Sal: saline solution, OV: vehicle, SS: silver sulfadiazine, LE 5: *Strychnos pseudoquina* 5%; LE 10: *S*. *pseudoquina* 10%. Data represented as mean ± SD. *,^†^ p<0.05, statistical difference between treatments: * vs. Sal and OV, *^†^ vs. Sal, OV and SS (Kruskal-Wallis test).

**Fig 3:** Representative photomicrographs obtained under polarizing microscopy demonstrate the distribution of collagen fibers in the scar tissue of rats treated with *Strychnos pseudoquina* ointment. Collagen fibers (type I) appear in shades of bright colors ranging from red to yellow, while thin reticular fibers (collagen type III) appear bright green. Tissue fragments were collected every 7 days during 21 days of treatment. Day 0 refers to the normal untreated tissue. Bar = 40 μm. Sirius red.

### Cytokine expression result

The TGF-β concentration was higher in the LE5, LE10 and SS than in the Sal and OV treatments on days 7 and 14. However, on day 14, TGF was higher in the LE group when compared to all other groups (Fig 4A). In relation to IL-10, the EL5 and EL10 groups presented increased values on the seventh day, when compared to the other groups (Fig 4B). TNF-α values were similar for all the groups (Fig 4C).

The article "Strychnos pseudoquina modulates the morphological reorganization of the scar tissue of second intention cutaneous wounds in rats" was retracted in 2025. Reasons: duplicated images; overlap with earlier publications; original data or images not available; concerns about the images.

**Fig 4:** Levels of transforming growth factor beta (TGF-β), Interleukin 10 (IL-10) and tumor necrosis factor (TNF-α) in scar tissue of rats treated with *Strychnos pseudoquina* extract. F1: treated tissue after seven days, F2: treated tissue, after 14 days. Sal: saline solution, OV: vehicle, SS: silver sulfadiazine, LE 5: *S*. *pseudoquina* 5%; LE 10: *S*. *pseudoquina* 10%. Data represented as mean ± SD. *^†^ p<0.05, statistical difference between treatments: * vs. Sal and OV, *^†^vs. Sal, OV and SS (Kruskal-Wallis test).

### Biochemical results

The MDA values were similar for all the groups (Fig 5A). The concentration of carbonylated proteins of animals from the LE5 and LE10 treatments was lower on day 14 (Fig 5B).

**Fig 5:** **Levels of malondialdehyde (MDA) (A), carbonylated proteins (PCN) (B), superoxide dismutase (SOD) (C) and catalase (CAT) (D) in scar tissue from rats treated with *Strychnos pseudoquina* extract**. F0: untreated normal tissue, F1: treated tissue after seven days, F2: treated tissue, after 14 days, F3: tissue treated after 21 days. Sal: saline solution, OV: vehicle, SS: silver sulfadiazine, LE 5: *S*. *pseudoquina* 5%; LE 10: *S*. *pseudoquina* 10%. Data represented as mean ± SD. *^†^ p<0.05, statistical difference between treatments: * vs. Sal and OV, *^†^ vs. Sal, OV and SS (Kruskal-Wallis test).

The levels of the enzyme superoxide dismutase (SOD) were higher in the treatments with LE, at concentrations of 5 and 10%, compared to Sal, OV and SS, on days 14 and 21 (Fig 5C). The catalase enzyme levels were higher with plant extract (LE5 and LE10) on the seventh day (Fig 5D).

## Discussion

The high proportions of flavonoid and alkaloid phenolic constituents in the *S*. *pseudoquina* extract indicate their healing effects. These molecules are bioactive for the treatment of health disorders [7,43], with antioxidant [44,45] and regenerative [46] abilities, as reported for polyphenols of *Dioclea violacea*, *Erythroxylum numularia* [47], *Brassica oleracea* [48] and *Bathysa cuspidata* [31]. We believe that plant research is a promising tool for the discovery of extracts or bioactive molecules that can contribute to the treatment of various diseases.

The higher rate of wound closure for those treated with *S*. *pseudoquina* based ointment indicates the activity of its components on cell proliferation, protein synthesis [49] and cell differentiation. This is a promising therapy, since it reduces the risk of complications. The area and wound closure speed describe the evolution of the wound [50]. Similar results were found in the topical treatment of wounds using essential oil from *Rosmarinus officinalis* in diabetic rats that presented higher wound contraction rate in 15 days of treatment. Similarly to the *S*. *pseudoquina* extract, this oil is rich in flavonoids, which may explain its high healing power.

The article "Strychnos pseudoquina modulates the morphological reorganization of the scar tissue of second intention cutaneous wounds in rats" was retracted in 2025. Reasons: duplicated images; overlap with earlier publications; original data or images not available; concerns about the images.

The higher number of mast cells found in our study in animals treated with LE extract, mainly LE10%, is important for the inflammatory phase of the scarring process, given that, when activated, they release chemical mediators that promote vasodilation and, consequently, cell migration [51,52]. These cells are important in the defense against pathogens [53], and present direct activity on the three phases of the scarring process [54], mainly the inflammatory stage. For Iba et al., [55], during the late phase of healing, a high number of mast cells on the edge of the wound stimulate the organization of collagen and help the remodeling of the tissue. Mast cells also promote the recruitment of neutrophils after an injury. Their absence is related with low number of cells and delayed healing process [56].

The higher proportion of collagen and elastic fibers in the treatments with *S*. *pseudoquina* confirms the faster rate of wound closure and the efficacy of the plant extract in the formation of a strong, resistant scar. Collagen plays a key role in skin healing, forming, and granulation tissues rich in collagen III at the beginning of the process, which serves as a framework for the deposition of collagen I, with thicker fibers that establish covalent bonds [57]. This architecture increases the resistance of the wound and, the greater the predominance of collagen I, the higher the maturation, firmness, and stiffness index of the newly formed tissue [33,58,59].

Our findings show increased TGF and IL-10 after treatment with LE extract. We believed that skin mast cells play a fundamental role in the regulation of inflammation due to the secretion of chemical mediators, mainly in the production of anti-inflammatory molecules that work directly on the resolution of inflammation by promoting cell proliferation, differentiation, migration and tissue remodeling [60]. TGF-β and IL-10 are considered universal mediators that can be synthesized by different cells, with positive action in the cutaneous repair process due to their capacity to accelerate matrix synthesis and tissue remodeling [61,62]. The results of our study corroborate this proliferative and remodeling effect, since the groups that received *S pseudoquina* extract showed increased amount of collagen and predominance of type I fibers, which give the tissue strength and resistance.

Similar values of malondialdehyde (MDA) between treatments indicate that S pseudoquina extract does not inhibit tissue oxidation. MDA is a byproduct of lipid peroxidation, derived from the breakdown of polyunsaturated fatty acids (linoleic, arachidonic and docosahexoic acid), considered the general biomarker of lipid oxidative damage in plasma [63] and the general potential biomarker of oxidative stress [64]. However, MDA is a very unstable molecule andthus the results obtained by the marking of this product are not completely reliable. Therefore, we can highlight the protein oxidation whose markers are carbonylated proteins. The higher the number of this marker, the greater the destruction of the tissue proteins by the activity of free radicals. When the tissue is damaged by the action of radicals, it is common to observe lipids, proteins, and cell DNA alterations, which lead to an oxidative stress [65]. In our study, the groups treated with extract presented lower PCN levels on the fourteenth day; this indicates that the extract protected the tissue from the action of free radicals. This may be due to the presence of the flavonoids and phenolic compounds found in the extract of *S*. *pseudoquina*. Similar studies with different medicinal plants have demonstrated the presence of isolated compounds, such as tannic acids and flavonoids, which showed significant antioxidant activity [66].

The article "Strychnos pseudoquina modulates the morphological reorganization of the scar tissue of second intention cutaneous wounds in rats" was retracted in 2025. Reasons: duplicated images; overlap with earlier publications; original data or images not available; concerns about the images.

The highest enzyme superoxide dismutase (SOD) levels in the treatments LE at 5 and 10% on days 14 and 21 indicate the stimulation of the cell antioxidant response by the *S*. *pseudoquina* extract. SOD is a component of the antioxidant cell system that promotes wound healing [67–68] and prevents the harmful effects of free radicals and other reactive oxygen species (ROS). This enzyme may be related to the presence of alkaloids, whose antioxidant activity was observed in the gastric ulcers of rats, by fraction of methanolic extract of *S*. *pseudoquina* enriched alkaloids, owing to efficient SOD production [29]. The higher levels of catalase enzyme (CAT) in treatments using *S*. *pseudoquina* extract (LE5 and LE10), on day seven of the experiment, show the antioxidant effect of this extract, since CAT is part of the cell antioxidant defense and catalyzes the decomposition of Hydrogen peroxide (H_2_O_2_) [15,69]. The topic treatment with *Phaleria macrocarpa* extract provided similar results, namely, increased SOD and CAT enzyme activity, reduced MDA levels and tissue damage, and accelerated wound healing processes [70].

## Conclusion

Our results indicate that *S*. *pseudoquina* extract has potential to heal cutaneous wounds in rats seven, 14 and 21 days after injury, and that they are more effective than silver sulfadiazine. This extract provides qualitative and quantitative benefits to the healing process by modulating the morphology of the damaged tissue, an additional mechanism through which it works during the initial phases of the tissue repair process in skin wounds. The healing effects were partially related to the ability of the topical treatment to stimulate cellularity, TGF-β and IL-10 levels, collagen, and elastic fibers deposition and attenuate oxidative damage in scar tissue, which accelerates wound closure. Additional studies involving different concentrations of LE and further analyses are needed for a more detailed definition of the molecular basis associated with the mechanism of action and applicability of this vegetable product as a viable therapeutic strategy in the treatment of cutaneous affections.
